RETRACTED

# Application Evaluation of High-Flow Humidified Oxygen in Patients with Respiratory Failure after General Anesthesia Extubation for Multiple Injuries

**DOI:** 10.1155/2021/1387129

**Published:** 2021-08-12

**Authors:** Ruijuan Ci, Yanjun Qin, Caizhe Ci, Chunhua Zhang, Shimin Dong, Mei Li

**Affiliations:** ^1^Department of Emergency Medicine, The Third Hospital of Hebei Medical University, Shijiazhuang, Hebei Province, China; ^2^Department of Cardiology, The Third Hospital of Hebei Medical University, Shijiazhuang, Hebei Province, China

## Abstract

**Objective:**

To explore the effect of high-flow humidified oxygen therapy (HFNC) on patients with respiratory failure after general anesthesia extubation for multiple injuries.

**Methods:**

214 patients with multiple injuries in our hospital who underwent general anesthesia and suffered respiratory failure after weaning extubation and received sequential treatment were included. And, they were divided into control group (HFNC group) and observation group (NIMV group) according to the random number table method. Patients in the control group (125 cases) used high-flow nasal cannula (HFNC) after general anesthesia extubation, while patients in the observation group (89 cases) used NIMV. The respiratory rate, heart rate, finger pulse oxygen, oxygenation index (PaO_2_/FiO_2_), and re-tracheal intubation rate in the two groups were compared at 2, 8, and 24 hours after sequential treatment, and the mortality rate and hospital stay of ICU time were whole-course observation. And, the effect of conventional oxygen inhalation or HFNC on oxygenation and prognosis was analyzed. Then, SPSS21.0 software was applied for statistical analysis. To analyze the effect of conventional oxygen inhalation or HFNC on the improvement of oxygenation and prognosis, the receiver operating characteristic (ROC) curve can be used to evaluate the feasibility and treatment effect of high-flow nasal oxygen therapy (HFNC) for patients with respiratory failure after general anesthesia extubation for multiple injuries.

**Results:**

Compared with the NIMV group, the respiratory frequency and heart rate of the HFNC group were significantly improved after 2 h, 8 h, and 24 h. At the same time, the finger pulse oxygen and oxygenation index increased significantly and returned to normal levels. HFNC can significantly reduce the reintubation rate, ICU hospital stay, and mortality rate. The area under the ROC curve was 0.9102, with 95% CI (0.8256, 0.9949) and *P* < 0.0001.

**Conclusion:**

For patients with multiple injuries undergoing general anesthesia and respiratory failure after weaning and extubation, the application of HFNC can moderate patients' heart rate and respiratory rate faster, increase oxygenation index and finger pulse oxygen, and reduce the reintubation rate, mortality rate, and ICU stay. At the same time, it can effectively improve the respiratory failure of patients after extubation and reduce the occurrence of complications.

RETRACTED

## 1. Introduction

Multiple injuries refer to traumas to 2 or more organs and anatomical parts caused by a single injury [1]. The condition is complex, and the fatality rate is high. Most of them require urgent surgical treatment. Intraoperative general anesthesia is the most routine anesthesia method in operation [2]. And, the anesthesia method needs to be selected according to the patients' condition, trying our best to avoid the inhibition of circulation, breathing, and liver and kidney functions, thereby affecting the patients' curative effect [3].

Respiratory failure is one of the serious complications after general anesthesia, and its incidence is as high as 3% [4]. Respiratory failure is the dysfunction of pulmonary ventilation and ventilation caused by various reasons, which can lead to an inability to carry out effective gas exchange, leading to hypoxia with carbon dioxide retention, which leads to a series of clinical synthesis of physiological and metabolic disorders [5, 6]. Postoperative hypoventilation is one of the key causes of respiratory failure after general anesthesia, and upper abdominal surgery and chest surgery are more serious [7, 8]. Supplemental oxygen is one of the first-line treatment methods for acute respiratory failure. Upper respiratory tract humidification and artificial respiration technology are not suitable for patients with dyspnea, which will cause discomfort and pain to patients [9, 10]. At the same time, dry, low-temperature high-flow oxygen will cause upper respiratory tract dryness and affect the comfort that the patients feel [10, 11].

High-flow humidified oxygen therapy and other oxygen therapy modes have significant advantages. Respiratory failure in patients after general anesthesia is caused by insufficient ventilation [12]. Low-flow oxygen therapy cannot effectively solve this problem. At the same time, the heating and humidification method can improve the clarity of lung mucus cilia in patients with bronchiectasis [13, 14]. Studies have shown that heating and humidification can improve the effect of oxygen treatment and reduce the complications of dryness. In summary, this article will analyze the application prospects of high-flow humidified oxygen therapy by analyzing the effect of this on respiratory failure after general anesthesia, to expand the application scope of high-flow humidified oxygen therapy.

RETRACTED

## 2. Materials and Methods

### 2.1. Research Object

Two hundred fourteen patients with multiple injuries who were treated in our hospital from December 2019 to February 2021 were selected. All patients experienced respiratory failure after general anesthesia extubation. The sequential treatment mode aims at infections caused by multiple injuries. Patients with multiple injuries all have the same injury factor causing 2 or more anatomical injuries, the patients' breathing state is relatively stable before treatment, and there is no symptom of respiratory failure. The patients were randomly divided into two groups, the control group (HFNC group, 125 cases) and the observation group (noninvasive mechanical ventilation group, 89 cases). In the noninvasive mechanical ventilation group, the ventilation was assisted through a noninvasive mechanical ventilator (NIMV) and the flow of oxygen was analyzed through a flow meter. The inhaled oxygen concentration was 40∼60% [15]. Continuous positive air pressure was 5∼8 cm H_2_O, the inspiratory pressure was 12∼18 cm H_2_O [16], and the air bubble humidifier increases humidity. Because the air bubble humidifier consists of cold water, the humidification effect is very limited. This is the most popular way of oxygen supply these days. The oxygen concentration for high-flow oxygen inhalation is 40%∼60%, the heating temperature is 37°C, and the oxygen flow rate is 40–60 L/min [17]. All patients have the right of informed consent, and this study has been approved by the Ethics Association of our hospital.

### 2.2. Diagnostic Criteria

After the patients were extubated from the ventilator after general anesthesia, respiratory failure occurred after spontaneous breathing of 30 min–1 h. After clinical hemogram analysis, the patients' signs of hypotension are still difficult to correct after adequate fluid supplementation. General systolic blood pressure (SBP) ≤90 mmHg, mean arterial pressure (MAP) <70 mmHg, SBP drop is greater than 40 mmHg, respiratory rate >30∼35 times/min, arterial blood gas conforms to the diagnosis of respiratory failure, and oxygenation index <200 mmHg [18, 19].

### 2.3. Design of Research

Patients randomly received standard oxygen therapy or HFNC. After sequential treatment, the respiratory rate, heart rate, finger pulse oxygen, oxygenation index (PaO_2_/FiO_2_), and reintubation rate were compared at 2, 8, and 24 hours. The mortality rate and ICU stay time were whole-course observation. And, the effect of conventional oxygen inhalation or HFNC on patients' oxygenation and prognosis was analyzed.

### 2.4. Statistical Analysis

All data were statistically analyzed by SPSS21.0, qualitative data were described as numbers (%), continuous data were expressed as mean ± standard deviation (*X* ± SD), and the range of nonnormally distributed data were expressed with median and quartile, and the nonparametric Mann–Whitney U test was used to compare variables. Categorical variables were analyzed by the Chi-square test and Fisher's test for small samples. *P* < 0.05 was considered statistically significant.

RETRACTED

## 3. Results

### 3.1. General Clinical Data

From December 2019 to February 2021, 214 patients with multiple injuries who were treated in our hospital were selected and suffered respiratory failure after general anesthesia extubation. According to different treatment methods, there were 125 cases and 89 cases in the high-flow oxygen inhalation group and the noninvasive mechanical ventilation group, respectively. And, the difference in the general statistics was not statistically significant. In the high-flow oxygen inhalation group, there were 64 males and 61 females, aged 45–78 years, with an average age of 62.45 ± 12.34 years, an average arterial pressure of 55.4 ± 5.3 mmHg, a respiratory frequency of 42.5 ± 6.4 times/minute, and an average oxygenation index of 168 ± 15.4 mmHg. In the noninvasive respiratory group, there were 46 males and 43 females, aged 43–81 years, with an average age of 61.51 ± 13.21 years, an average arterial pressure of 56.2 ± 4.8 mmHg, a respiratory frequency of 45.2 ± 5.4 times/minute, and an average oxygenation index of 165.8 ± 17.4 mmHg. The differences in the general statistics of patients in the two groups were not statistically significant (*P* > 0.05), as can be seen in Table 1.

### 3.2. Comparison of Reintubation Rates between the Two Groups

During the treatment, the patients have persistent hypoxia that cannot be corrected, respiratory muscle fatigue, a Glasgow score of consciousness disturbance <12 points, increased airway secretions, difficulty in expectoration, unstable hemodynamics, and arterial blood gas pH ≤ 7.30. 3 cases were reintubated in the HFNC group and 8 cases were reintubated in the NIMV group, accounting for 10.0% and 27.6%, respectively, with *P* < 0.05, as shown in Figure 1.

### 3.3. Changes in Respiratory Frequency and Heart Rate of Patients in the Two Groups

The changes of the respiratory frequency and heart rate of patients in the two groups area observed at 2 h, 8 h, and 24 h after the treatment. The HFNC group can return to the normal heart rate faster than the NIMV group, and the difference is statistically significant at 2 h and 8 h, with *P* < 0.05. The reduction of respiratory frequency was more significant in the HFNC group. The respiratory frequency of patients in the HFNC group was significantly lower than that in the NIMV group at 8 h and 24 h and was closer to the normal respiratory rate, *P* < 0.05, as shown in Figure 2.

RETRACTED

### 3.4. Changes in Finger Pulse Oxygen and Oxygenation Index in the Two Groups

The finger pulse oxygen (75.0% ± 3.5) increased significantly in the HFNC group at 2 h, which was statistically significant compared with the NIMV group (66.6 ± 4.2), with *P* < 0.05; at 8 h (94.3% ± 3.2) and 24 h (98.2% ± 1.2), finger pulse oxygen concentration was higher than in the NIMV group (83.2% ± 3.2, 94.4% ± 4.5) and returned to a relatively normal level. The difference was statistically significant, with *P* < 0.05; the oxygenation index of the HFNC group at 2 h, 8 h, and 24 h increased significantly, compared with the NIMV group, and the difference was statistically significant, as shown in Figure 3.

### 3.5. Mortality Rate and ICU Stay in the Two Groups

The mortality rate of the HFNC group was 6.4% (8/125), while the mortality rate of the NIMV group was 28.1% (25/89). The mortality rate of the NIMV group was significantly higher than that of the HFNC group, with *P* < 0.05, as can be seen in Table 2. The average ICU stay of patients in the NIMV group (78.4 ± 12.3 h) was significantly longer than in the HFNC group (45.5 ± 8.6 h), and the difference was statistically significant, with *P* < 0.05, as can be seen in Table 2.

### 3.6. ROC Curve Is Divided into Two Groups of Patients to Improve Oxygen and Index

Taking the 8 h oxygenation index as the evaluation and analysis standard, compared with the NIMV group, the area under the curve in the HFNC group was 0.9102, with 95% CI (0.8256, 0.9949) and *P* < 0.0001, as shown in Figure 4.

## 4. Discussion

It is common to acquire multiple organ dysfunctions after multiple injuries, and the lungs are the first organs that are affected, often leading to acute respiratory failure and extremely high mortality. Mechanical ventilation after general anesthesia extubation is an important clinical technique for patients with multiple injuries to support breathing and maintain life [20].

High-flow warming and humidifying nasal catheter oxygen therapy is a new type of oxygen therapy method [20, 21]. The modified oxygen therapy system is mainly composed of an air-oxygen mixing valve, heating humidifier, and heating wire [22]. The heating and humidifying oxygen or air-oxygen mixed gas is transmitted through the catheter. Oxygen therapy can supplement the patients with oxygen, increase the patients' arterial blood oxygen partial pressure (PaO_2_) and arterial blood oxygen saturation (SaO_2_), treat patients with hypoxia caused by various factors, increase the metabolic process, and promote the body to perform normal life activity [23].

RETRACTED

That high-flow humidification oxygen therapy can significantly reduce the mortality and the stay time in ICU, effectively save the patients' lives, and reduce the financial burden has been found in research. Comfortable oxygen therapy methods are beneficial to improve the patients' treatment compliance and enhance the treatment effect. At the same time, high-flow warming and humidifying oxygen therapy have a good tracheal channel humidification effect, and the relative humidity is maintained at about 100%, keeping the upper respiratory tract mucosa from being damaged, and the cilia can move normally, thereby clearing the respiratory tract excrement [24].

In the study, it was found that compared with traditional oxygen therapy, high-flow humidified oxygen therapy has the advantage of rapidly increasing finger pulse oxygen and oxygenation index in the effect of respiratory failure in patients with multiple injuries after extubation. It can significantly increase the patients' finger pulse oxygen and oxygenation index at 2 h after treatment, thereby saving the patients' life. The traditional oxygen therapy method has the shortcoming of slow effect, and it is easy to withdraw the tube again and even end the patients' life. Regarding the effect of high-flow humidified oxygen on the respiratory frequency and heart rate, due to early respiratory failure, airway obstruction, and rapid breathing rate, high-flow humidified oxygen can significantly improve this situation, thereby reducing the patients' rapid breathing rate and the abnormal heart rate, which can make patients recover better [25, 26].

The heating and humidification of the artificial airway and tube channel will be an important content of oxygen therapy for patients with multiple injuries after weaning. The establishment of a good airway channel directly affects the patients' therapeutic effect, and high-flow oxygen therapy has a good humidification effect and improves the patients' treatment comfort, enhancing the patients' treatment compliance and treatment effect.

## Figures and Tables

**Figure 1:** Frequency of reintubation of patients in the two groups; ^*∗*^the difference between the two groups is statistically significant, *P* < 0.05.

**Figure 2:** Changes in heart rate and respiratory frequency of patients with respiratory failure in the two groups after different treatments; ^*∗*^*P* < 0.05.

**Figure 3:** Changes in finger pulse oxygen and oxygenation index of patients in the two groups; ^*∗*^*P* < 0.05.

**Figure 4:** ROC curve.

**Table 1:** Comparison of general information of patients in the two groups.

Group	*N*	Male/female (n)	Age	MAP (mmHg)	RR	OI (mmHg)
HFNC	125	64/61	62.45 ± 12.34	55.4 ± 5.3	42.5 ± 6.4	168 ± 15.4
NIMV	89	46/43	61.51 ± 13.21	56.2 ± 4.8	45.2 ± 5.4	165.8 ± 17.4

RETRACTED

**Table 2:** Mortality rate and ICU stay in the two groups.

Group	*N*	Mortality	ICU (h)
HFNC	125	6.4%	45.5 ± 8.6
NIMV	89	28.1%^*∗*^	78.4 ± 12.3^*∗*^

*Note*. ^*∗*^*P* < 0.05 compared with the HFNC group.

## Data Availability

The data used to support the findings of this study are included within the article.
